The article "Experimental research on rapid removing characteristics of carbon monoxide generated during gas explosions" was published in 2022. Journal: PLoS One.

# Experimental research on rapid removing characteristics of carbon monoxide generated during gas explosions

**DOI:** 10.1371/journal.pone.0267553

**Published:** 2022-05-04

**Authors:** Yashengnan Sun, Xihua Zhou, Ang Li, Gang Bai, Tianyu Xin, Jue Wang, Mufeng Xiao

**Affiliations:** 1 College of Safety Science and Engineering, Liaoning Technical University, Fuxin, China; 2 Key Laboratory of Mine Thermodynamic Disaster and Control of Ministry of Education, Huludao, China; 3 School of Safety Engineering, North China Institute of Science and Technology, Beijing, China; 4 Institute of Mechanics and Engineering, Liaoning Technical University, Fuxin, China; 5 College of Civil Engineering, Liaoning Technical University, Fuxin, China; 6 College of Architecture and Transportation, Liaoning Technical University, Fuxin, China; Universiti Malaysia Pahang, VIET NAM

## Abstract

A large amount of gas, such as CO, accumulates in a coal mine after an explosion, leading to CO poisoning. In this study, a self-developed platform was used to eliminate CO from coal mines and determine the mass of the rapidly eliminated CO and its concentration in the eliminated gases. Equations were derived to calculate the amount of CO eliminated and the removing rate. The results showed that a rapid removing reagent in the form of nonprecious metal catalysts is useful for removing CO. Removing agents with larger masses facilitated the activation, irrespective of the CO concentration. For removing reagent amounts of 10, 15, 20, 25, and 30 g, the amount of CO eliminated, the removing rate, and the time required to complete catalytic oxidation increased sequentially. The CO removing process could be divided into three stages (I, II, and III) based on the variations in the CO, CO_2_, and O_2_ concentrations during CO removing. The removing reagent first chemically adsorbs CO and O_2_, and then desorbs CO_2_. The final CO concentration tends to 0, the O_2_ concentration remains stable, and the CO_2_ concentration decreases. This shows that the ablation agent has an impact on the changes in the CO and CO_2_ concentrations.

## 1 Introduction

Coal is the main energy in China [1–5], accounting for 56.8% of the primary energy production and consumption institutions. In the process of coal mining, the underground space of coal mine is relatively closed, and the poorly ventilated area is easy to accumulate CO [4, 6, 7], leading to the deterioration of internal air quality. After inhalation, CO is easy to combine with hemoglobin in the blood, forming carbon oxygen hemoglobin (COHb) to weaken the oxygen carrying capacity of hemoglobin, resulting in the death of underground personnel asphyxiation. After the gas explosion, the oxygen concentration in the air of underground coal mine drops rapidly, and a large amount of CO gas is produced, which leads to the change of atmospheric composition in the roadway [2]. About 70–80% of underground people die from CO poisoning in gas or coal dust explosion accidents [4]. CO eliminator was prepared and CO was catalyzed to CO_2_ by catalytic oxidation method to rapidly reduce the concentration of CO [8, 9]. The CO_2_ produced has a certain effect of 3 gas explosion to ensure the safety of downhole personnel to the greatest extent.

In recent years, the CO catalysts has been extensively studied. Njagi et al. developed metal oxides and studied their catalytic oxidation performance for CO. Cimino [10] synthesized Pt nanoparticles to cover the surface of CeO_2_ catalyst, which improved the catalytic oxidation activity of CO and increased the stability of its catalytic oxidation. Chun-Wan Yen [11] prepared a new type of Au–Ag bimetallic nanocatalyst supported on a mesoporous silicon carrier, which exhibited a high activity and stability and did not deactivate in a humid environment. Ching-Shiun Chen [12] studied the oxidation of CO on Cu/TiO_2_ catalysts with different Cu loadings. Xianglan Xu [13] prepared a series of Sn-modified Co_3_O_4_ catalysts with different Co/Sn molar ratios using the co-precipitation method. The results showed that adding a small amount of Sn to Co_3_O_4_ had little effect on its CO oxidation activity, but significantly improved its water resistance.

Most existing research on development, characterization [14–29], and basic performance comparison of different catalysts of CO catalyst [17, 29–31]. A single-catalyst characterization and performance comparisons cannot fully reflect the CO ablation effect in a coal mine. Understanding the influences of the removing agent quantity and CO concentration on the ablation performance is of great significance to the practical application of removing agents in coal mines. To this end, we applied an independently developed CO ablation experimental platform to study the effects of removing agent quantity and CO concentration on the ablation performance and ablation process. New removing agent characterization indicators were derived, and the CO removing volume and removing rate were determined. The rate calculation method was used to analyze the quantitative relationship between the removing volume, removing rate, removing agent quantity, and CO concentration. The results of provide a theoretical help for its rapid removing in the unfortunate event of gas explosions.

## 2 Experimental methods

### 2.1 Removing agent

CO is accumulated following a gas explosion in a coal mine. Because the ventilation equipment is seriously damaged, an efficient CO ablation is vital to the safety of personnel. CO catalysts can be mainly divided into two categories: nonprecious metal catalysts and precious metal catalysts. Noble metal catalysts have good catalytic effects but are expensive. Considering economic factors, we used nonprecious metal catalysts as removing agents in our experimental research. The widely used nonprecious metal catalysts in China are Cu-supported catalysts. Cu^+^ forms a complex with CO molecules, which is selective for CO catalysis [32]

For the experiment, a nonprecious metal catalyst was selected. N_2_ adsorption and desorption were employed to test the specific surface area of the sample; S_BET_ = 179.2016 m^2^·g^−1^. Fig 1 shows a sample of the removing agent and the sample preparation process.

**Fig 1:** A sample of the removing agent and the sample preparation process.

### 2.2 Experimental scheme

Fig 2 shows the experimental device. The experimental device:

1. Gas distribution system, including gas cylinders and pressure gauges.
2. Ablation system, including a test tank and a reaction chamber.
3. Temperature and pressure data acquisition system, including temperature sensors, pressure sensors, and paperless recorder. Table 1 shows the experimental instrument parameter.
4. Gas analysis system, comprising a condenser and a gas analyzer.
5. Exhaust system, including vacuum pumps and exhaust pipelines.

**Fig 2:** Schematic of the experimental system developed for CO gas ablation.

**Table 1:** Experimental instrument parameter.

Instrument	Model	Range	Precision	Manufacturer
Temperature sensor	Pt100	−50–200°C	0.1%FS	-
Pressure sensor	-	0–2.5000 MPa (absolute pressure)	0.5%FS	Yantai Asustek precision equipment
18-channel paperless recorder	MIK-R9600	-	-	Hangzhou Meacon Automation Technology Co., Ltd
Gas analyzer	Infrared CO sensor	0–10%	2%FS	Shenzhen Sunike Technology Co., Ltd.
	Infrared CO_2_ sensor	0–20%	2%FS	
	Electrochemical O_2_ sensor	0–25%	3%FS	

The gas analyzer was used for the gas analysis, in conjunction with a condenser. The condenser was employed to condense the gas to temperatures below 5°C and dry it.

### 2.3 Experimental program

For the experimental program, we employed high-purity CO (99.999%), O_2_ (99.999%), and N_2_ (99.99%) to prepare the gas. Since the highest CO generated after a gas explosion is 8% [8], a mixed gas with a CO concentration of 5% was prepared according to Dalton’s law of partial pressure, and the mass of the removing agent was set to 10, 15, 20, 25, and 30 g. Based on the experimental results, 15 g of the agent was selected, and the CO concentration was set to 1%, 3%, 5%, and 7%.

The removing object was CO gas in the removing system, the test tank volume was 1884 cm^3^, the reaction chamber volume was 300 cm^3^, and the total removing volume was 2184 cm^3^.

After placing a certain quantity of the removing agent in the reaction chamber, a mixed gas at a pressure of 0.12 MPa was sent to the test tank. After the gas analyzer was stabilized, the reaction chamber value was opened. At this time, the pressure was approximately 0.1 MPa; the test tank, reaction chamber, and gas analysis system formed an internal loop to test and record the changes in the CO, CO_2_, and O_2_ concentrations in the test tank and reaction chamber. Thus, we explored the effects of the quantity of the removing agent and CO concentration on the removing performance, and analyzed the removing process.

The specific experimental steps were as follows:

1. Air tightness inspection: The experimental system was inspected for air tightness.
2. Vacuum. The experimental system was vacuumed until the pressure remained stable (approximately −0.0994 MPa).
3. Gas distribution. Based on the gas injection pressure readings listed in Table 2, gas distribution was carried out, where N_2_, O_2_, and CO gases were injected.
4. Placement of removing agent. An electronic balance was used to weigh 10, 15, 20, 25, and 30 g (accurate to 0.01 g) of the removing agent. After weighing, the removing agent was placed in a reaction bag, which was then placed in the reaction chamber, for the experiment.
5. Constant temperature. To ensure that the temperature of each tank was consistent, a water bath and heating belt were used to keep the temperature of the experimental system constant at 25°C.
6. The removing system was vacuumed.
7. Test. The gas analysis system valve was opened, and the mixed gas was passed through the gas analyzer until the indicator was stable. We then opened the reaction chamber valve, and monitored and recorded the changes in the O_2_, CO, and CO_2_ concentrations in the loop.
8. Exhaust. The gas was exhausted from the test tank and reaction chamber through the exhaust port and evacuated to ensure that there was no CO residue in the removing system. Since the lowest CO concentration allowed for people under normal working conditions is 24 ppm, which is 0.0024%, when the CO concentration was reduced to 0 in the experiment, it was considered that the lowest allowable CO concentration was reached, and the experiment was terminated at this time.

**Table 2:** Pressure during gas injection.

No.	CO concentration (%)	O_2_ concentration (%)	N_2_ concentration (%)	Absolute pressure /MPa	Pressure after N_2_ injection /MPa	Pressure after O_2_ injection /MPa	Pressure after CO injection /MPa
**1**	1	19.80	79.20	0.6	0.4752	0.5940	0.6000
**2**	3	19.40	77.60	0.6	0.4656	0.5820	0.6000
**3**	5	19.00	76.00	0.6	0.4560	0.5700	0.6000
**4**	7	18.60	74.40	0.6	0.4464	0.5580	0.6000

### 2.4 Removing performance indicators

After a coal mine gas explosion, the ventilation facilities are significantly damaged, the wind flow is turbulent, and harmful gases accumulate at the explosion location. The explosion area will be in a closed state. Two indicators, namely the removing volume and removing rate, are proposed to reflect the CO removing performance of the rapid removing agents under airtight conditions.

The experimentally obtained removing volume and removing rate were used to characterize the CO removing capability of the fast-acting removing agent. The removing volume is the amount of CO removed per unit mass of the removing agent after CO comes in contact with it. The volume and amount of removing can be used to evaluate removing performance. The higher the removing rate, the higher the removing performance.

The instantaneous removing rate refers to the amount of CO removing in unit time. The average removing rate is the volume of CO removing during the whole experiment, and the calculation formula for the removing amount is:

$$S=\frac{\left|\varphi^{\prime \prime }-\varphi^{\prime }\right|V}{m}$$ (1)

In the formula, *S* is the removing volume, cm^3^·g^−1^; *φ”* and *φ’* is the concentration of CO at the time of experiment t_2_ and t_1_, %; *V* is the volume of the system, cm^3^; *m* is the mass of the removing agent, g.

The formula for calculating the total removing volume is:

$$S_{T}=\frac{\left|\varphi_{2}-\varphi_{1}\right|V}{m}$$ (2)

where *S*_*T*_ is the total removing volume, cm^3^·g^−1^; *φ*_*2*_ and *φ*_*1*_ is the CO concentration at the end and beginning of the experiment, %.

The instantaneous removing rate calculation formula is:

$$v=\frac{dS}{dt}$$ (3)

where *v* is the removing rate, cm^3^·g^−1^·s^−1^; *t* is the time, s.

The formula for calculating the average removing rate is:

$$\bar{v}=\frac{\left|\varphi_{2}-\varphi_{1}\right|V}{t_{T}}$$ (4)

where *φ* is the average removing rate, cm^3^·s^−1^; *t*_*T*_ is the total time from the beginning to the end of the experiment, s.

## 3 Results and discussion

### 3.1 Experimental system

The removing system without the removing agent was evacuated and filled with the mixed gas at a pressure of 0.1013 MPa, in which the CO, O_2_, and N_2_ concentrations were 5%, 19%, and 76%, respectively. The tank temperature was controlled at 25°C, and there were no changes in the gas concentration nor any increase in the temperature as recorded by the temperature sensor under the experimental conditions. Therefore, only the effect of gas concentration and eliminator on activity can be considered in the experimental process.

### 3.2 Effect of removing reagent amount

Using Eq (1), the variation trends in the CO removing amount and the CO concentration over time are obtained, as shown in Figs 3 and 4.

**Fig 3:** Variation in the CO elimination amount over time (different elimination amounts).

**Fig 4:** Variation in the concentration of CO over time (different elimination amounts).

Fig 3 shows that the lower the mass of the removing agent, the greater the amount of CO removing. The curves of removing agents with different masses have different reaction times after entering the stable period of reaction. More specifically, removing agents with masses of 10, 15, 20, 25, and 30 g require 4522, 1217, 310, 244, and 235 s, respectively, to reach the maximum removing volume. The greater the quantity of the removing agent, the shorter the response time. The greater the amount of removing agent, the greater the number of surface active sites and the shorter the reaction time.

The CO concentration directly affects the life and safety of underground personnel. The faster the reduction in the CO concentration to a safe value, the safer the underground personnel. Fig 4 shows that the effect of the removing agent quantity varies in the reaction catalysis period: the higher the quantity, the better the removing effect, consistent with a previous result [33]. When 5% CO was treated with 10 g of the rapid removing agent, the CO concentration reduced to 0.51% (5100 ppm), the reaction rate rapidly reduced, and the reaction time significantly increased. Removing agents with masses of 15, 20, 25, and 30 g could reduce the high CO concentration to 0.08% (800 ppm), 0.07% (700 ppm), 0.03% (300 ppm), and 0.03% (300 ppm), respectively, and then enter a stable period of the reaction when the gas concentration no longer changes. Based on these results, when using removing agents for CO removing after a gas explosion in coal mines, removing agents of different quantities can be placed at different locations.

Using Eq (3), the removing rate is calculated, as shown in Fig 5. Fig 5 shows that, the greater the removing agent quantity, the lower the peak removing rate, and the peak value is reached. The time required is less, and the rule is shown in Fig 6. The peak removing rates for removing agent masses of 10, 15, 20, 25, and 30 g are 0.42593, 0.34218, 0.23479, 0.14852, and 0.12013 cm^3^·g^−1^·s^−1^, respectively, and the times required to reach the peak are 77, 57, 51, 49, and 36 s, respectively. After the removing agent was activated, its activity was closely related to the number of CO molecules around it. The lower the mass of the removing agent, the greater the number of CO molecules around it, and the greater the amount of removing per unit time. The peak removing rate was inversely proportional to the mass of the removing agent. The greater the mass of the removing agent, the shorter the time required to reach the maximum removing rate. This is because, the greater the mass of the removing agent, the shorter the catalytic activation period, and the earlier it enters the catalytic reaction period, the shorter the time required to reach the maximum removing rate. Since the removing agent -catalyzed oxidation of CO conforms to the Mars–van Krevelen mechanism [33–36], the greater the mass of the removing agent, the higher the lattice oxygen content on its surface, thus reducing the catalytic activation period.

**Fig 5:** Variation in the CO elimination rate over time (different elimination amounts).

**Fig 6:** Variations in the peak elimination rate and time required to reach maximum elimination rate with the quantity of the elimination amount (different elimination amounts).

Using Eqs (2) and (4), the average removing rate and total removing volume of the CO removing with different removing agent quantities are calculated. Fig 7 shows that the average removing rate increases with the increase in the removing quantity. At higher removing quantities, the reaction catalysis period time is not much different; however, the reaction plateau time decreases as the removing mass increases. The reaction time also decreases as the mass of the removing agent increases, and the reaction rate increases accordingly. The average removing rates for removing agent masses of 10, 15, 20, 25, and 30 g were 0.0250, 0.0928, 0.3650, 0.4619, and 0.4796 cm^3^·s^−1^, respectively. For removing agent masses of 10 g and 15 g, the average removing rate was <0.1 cm^3^·s^−1^, and for masses of 20, 25, and 30 g, the average removing rate was >0.3 cm^3^·s^−1^. When the mass of the removing agent was increased from 15 g to 20 g, the removing rate increased significantly.

**Fig 7:** Variations in the average elimination rate and total elimination amount with the elimination reagent (different elimination amounts).

Fig 7 shows that the total amount of CO removing decreases with increasing mass. The total removing amounts for removing agent masses of 15, 20, 25, and 30 g are 11.3136, 7.5570, 5.6568, 4.5080, and 3.7567 cm^3^·g^−1^, respectively. This is because the CO removing process is a surface reaction. The greater the mass of the removing agent, the fewer the relative CO molecules on the surface, the higher the CO concentration, and the lower the removing of CO molecules per unit mass of the removing agent, the lower the removing amount.

### 3.3 Effect of CO concentration

The removing agent quantity was set to 15 g, and removing experiments with CO concentrations of 1.29%, 3.13%, 5.16%, and 7.69% were conducted.

The experiment was conducted in Liaoning, China, the season is winter, and the ambient temperature was as low as -20°C, resulting in low gas temperature. After gas distribution, the concentration of experimental gas was different from that of the designed gas, but the analysis of experimental results was not affected.

Using Eq (1), the CO removing volume was obtained. Figs 8 and 9 show the variation trends in the CO concentration and CO removing volume over time during the removing process.

**Fig 8:** Variation in the concentration of CO over time (different CO concentrations).

**Fig 9:** Variation in the CO elimination amount over time (different CO concentrations).

Fig 8 shows that when performing removing with different CO concentrations, there still exist a catalytic activation period, a catalytic reaction period, and a reaction plateau period. The CO concentration has no significant effect on the catalytic activation period, which is approximately 41 s. This shows that the time required for catalytic activation is only related to the quantity of the removing agent, irrespective of the CO concentration. When the removing agent quantity is the same, the activating components contained in it are the same, and the time required for CO to activate the removing agent is the same.

Different CO concentrations have different complete catalytic oxidation times. The higher the CO concentration, the longer it takes for complete oxidation. The complete catalytic oxidation times for CO concentrations of 1.29%, 3.13%, and 5.16% are 447, 670, and 1223 s, respectively. Fifteen grams of the removing agent cannot fully catalyze and oxidize 7.69% of CO in the removing system. This is because when the CO concentration is high, the removing system contains many CO gas molecules. The inability to completely ablate the CO molecules in the case of the 7.69% concentration is due to the supersaturation of the CO molecules. The activated components contained in the removing agent can ablate the CO molecules less than the CO molecules present in the mixed gas, and the CO molecules cannot be completely catalyzed and oxidized.

Figs 9 and 10 show that the peaks of the CO removing amount and CO concentration are proportional, and the fitting formula is *y* = 0.1441*x*+1.4032, and when the CO concentrations are 1.29%, 3.13%, 5.16%, and 7.69%, the peak removing volumes are 1.8783, 4.5721, 7.5133, and 10.8477 cm^3^·g^−1^, respectively. The higher the CO concentration, the greater the removing volume. This is because when the CO concentration is <7.69%, the removing agent mass is in a state of oversaturation, i.e., the ability to ablate CO is greater than the CO molecules in the removing system; therefore, the higher the number of CO molecules, the higher the removing amount and the greater the volume of CO ablated per unit mass. When the CO concentration is ≥7.69%, the mass of the CO molecules is in a state of supersaturation, and the CO molecules cannot be completed ablated. In the CO concentration range of 5.16%–7.69%, the masses of the CO molecules and removing agent are just saturated in a certain state, and the removing amount is maximum, 10.8477 cm^3^·g^−1^.

**Fig 10:** Peaks of CO elimination rate and elimination amount over time (different CO concentrations).

Figs 10 and 11 show that, the higher the CO concentration, the greater the removing rate. The principle of CO removing is the catalytic oxidation reaction, and the reaction is expressed in Eq (5).


$$2\mathrm{CO}+O_{2}\overset{\mathrm{Elimination}}{\Rightarrow }2{\mathrm{CO}}_{2}$$ (5)

**Fig 11:** Variation in the CO elimination rate over time (different CO concentrations).

When the CO concentration is high, the CO concentration per unit time decreases faster, and the CO_2_ concentration increases faster, i.e., when the response is faster, the greater the removing rate, the greater the corresponding peak removing rate. When the CO concentrations are 1.29%, 3.13%, 5.16%, and 7.69%, the peak removing rates are 0.0655, 0.1602, 0.3422, and 0.4295 cm^3^·g^−1^·s^−1^.

## 4 Removing process analysis

Taking the experiment where *m* (removing agent) = 20 g and c (CO) = 5% as an example, the gas composition of the removing process was analyzed. During the experimental reaction process, the test tank, the reaction chamber, and the connecting pipeline were considered rigid components and were tested for airtightness. The experimental reaction process was considered a constant-volume process, in which case, we have:

$$\frac{\Delta c_{1}}{\Delta c_{2}}=\frac{n_{1}}{n_{2}}=\frac{\eta_{1}}{\eta_{2}}$$ (6)

Fig 12 shows the trend in the concentrations of each gas over time during the experiment. At the beginning of the experiment, the CO concentration decreased rapidly, and the CO_2_ and O_2_ concentrations increased. Until 84 s, the oxygen concentration increased from the initial 21.22% to a maximum value of 22%. At this time, the CO_2_ concentration exhibited inflection point 1, at which the CO_2_ concentration was 0.58%; at this stage, the gas change for each concentration in Stage I was complete.

**Fig 12:** Variations in the O_2_, CO, and CO_2_ concentrations over time.

In the first stage, the CO molecules were first chemically adsorbed onto the surface of the removing agent, which raised the CO molecules to the first excited state [22], thereby increasing their chemical reactivity. While chemically adsorbing CO, the removing agent released a small amount of O_2_ molecules, which increased the oxygen concentration. At this time, the CO and O_2_ molecules accumulated in a large amount to generate CO_2_ molecules. The growth rate of CO_2_ during this period was higher than that in the later period.

After the first stage, CO was almost completely chemically adsorbed by the removing agent, and after the CO concentration drops to 0.37%, the chemical adsorption rate of CO by the removing agent dropped rapidly, and the amount of oxygen released decreased, thereby reducing the CO concentration on the surface of the removing agent, decreasing the reaction rate, and leading to a slower CO_2_ growth. At this time, the second stage of the reaction commenced. In the second stage, the O_2_ molecules produced were less than the consumed O_2_ molecules; therefore, the O_2_ concentration also began to decrease, the reaction rate reduced, and the CO_2_ concentration curve slowed down until the reaction was complete; at this point, inflection point 2 appeared.

In the second stage of the reaction, the change in the CO concentration was <0.37%, which was less than the initial concentration of 5%; therefore, the O_2_ released by the removing agent when chemically adsorbing CO was negligible. It is considered that the O_2_ consumed in the removing process was completely converted into CO_2_. In this case, Eq (6) can be solved as: $\frac{\Delta c_{O_{2}}}{\Delta c_{CO_{2}}}=\frac{n_{O_{2}}}{n_{CO_{2}}}=\frac{\eta_{O_{2}}}{\eta_{CO_{2}}}=\frac{1}{2}=0.5\frac{\Delta c_{O_{2}}}{\Delta c_{CO_{2}}}=\frac{n_{O_{2}}}{n_{CO_{2}}}=\frac{\eta_{O_{2}}}{\eta_{CO_{2}}}=\frac{1}{2}=0.5$

In Phase II, $\Delta c_{O_{2}}$ = 22%–20.26% = 1.74%. The change in CO_2_ generated theoretically is $\Delta c_{CO_{2T}}$ = 3.48%, but actually $\Delta c_{CO_{2_{A}}}$ = 3.42%–1.01% = 2.41%; $\Delta c_{CO_{2T}}-\Delta c_{CO_{2A}}$ = 1.07%

From the stoichiometric ratio,

$$\frac{\Delta c_{O_{2}}}{\Delta c_{CO_{2A}}}=0.72>0.5$$

This shows that a part of CO_2_ was adsorbed by the removing agent during the generation process, which was not completely tested.

After inflection point 2, the reaction entered the third stage. At this stage, the CO_2_ concentration curve appeared to decrease in a narrow range, whereas the O_2_ and CO concentration curves were relatively stable. This further shows that CO_2_ is not completely desorbed, and a further analysis of the CO_2_ concentration is required.

Fig 13 shows that the CO_2_ concentration produced under different removing agent quantities is different, and the greater the removing agent quantity, the lower the CO_2_ concentration, which again proves that the rapid removing agent has an adsorption effect on CO_2_. The quantity of the removing agent is different, and the time to enter inflection point 1 and the CO_2_ concentration are mostly different. For 10 g, the inflection point 1 is reached in 77 s, and the CO_2_ concentration is 1.26%. For 15 g, the inflection point 1 is reached in 89 s, and the CO_2_ concentration is 1.01%. Entering turning point 1, the CO_2_ concentration is 0.73%. When the removing agent mass is less than or equal to 20 g, the greater the mass of the removing agent, the longer it takes to reach inflection point 1 and the lower the CO_2_ concentration at inflection point 1.The removing process of the removing agent conforms to the Mars–van Krevelen mechanism [6]. The CO molecules first react with the lattice oxygen on the surface of the removing agent to generate CO_2_ molecules and desorb, then O_2_ supplements the lattice oxygen to generate adsorbed oxygen, and the CO molecules continue to adsorb oxygen. The reaction proceeds.

**Fig 13:** Variations in the CO_2_ concentrations over time (different elimination amounts).

## 5 Conclusions

To avoid suffocation and casualties due to CO poisoning in the event of a gas explosion in coal mines, a CO removing experiment was conducted using an independently developed experimental method. The conclusion is as follows:

1. Calculation methods for the removing volume and rate were put forward. Based on the growth rate of the removing volume, the removing process presented a “three-stage” characteristic: a catalytic activation period, a catalytic reaction period, and a reaction plateau period. The greater the mass of the removing agent, the easier the activation and the shorter the catalytic activation period, irrespective of the concentration.
2. The quantitative relationship between the removing volume and the removing rate and that between the removing agent quantity and CO concentration were analyzed. The greater the quantity of agent, the lower the removing volume and the higher the removing rate. The higher the CO concentration, the greater the removing volume and the higher the removing rate.
3. The process of CO removing using a rapid removing agent was studied. Based on the change in the gas concentrations, the removing process could be divided into three stages: I, II, and III. In Stage I, the CO concentration rapidly reduced because of the chemical adsorption on the surface of the removing agent, and small amounts of CO_2_ and O_2_ were produced. In Stage II, the theoretically calculated CO_2_ concentration was less than the actual value, indicating that the rapid removing agent had removing effects on both CO and CO_2_. In Stage III, the concentration curves of CO and O_2_ were stable, whereas the CO_2_ concentration decreased, further demonstrating that the removing agent had an effect on both the CO and CO_2_ concentrations.
4. The research results provide a theoretical basis for the fast removing of CO generated after a gas explosion, improve the economics of the use of removing agents, and reduce the occurrence of accidents that cause suffocation and casualties due to CO poisoning.

## Supporting information

S1 File (ZIP)
